The article "Posttreatment Recurrence and Death Patterns in Patients with Advanced Esophageal Cancer" was published in 2022. Journal: Dis Markers.

# Posttreatment Recurrence and Death Patterns in Patients with Advanced Esophageal Cancer

**DOI:** 10.1155/2022/1094597

**Published:** 2022-07-09

**Authors:** Xiangmei Zhang, Hui Wang, Dongwei He, Ming He, Xin Chen, Jidong Zhao

**Affiliations:** ^1^Research Center, Fourth Hospital of Hebei Medical University, Shijiazhuang 050011, China; ^2^Hebei Provincial Key Laboratory of Tumor Microenvironment and Drug Resistance, Hebei Medical University, Shijiazhuang 050017, China; ^3^College of Life Sciences, Hebei Normal University, Shijiazhuang 050024, China; ^4^Laboratory of Pathology, Hebei Cancer Institute, The Fourth Hospital of Hebei Medical University, Shijiazhuang, China; ^5^Department of Thoracic Surgery, Fourth Hospital of Hebei Medical University, Shijiazhuang 050011, China

## Abstract

**Objective:**

To investigate into the clinical factors associated with posttreatment recurrence and death patterns in patients with advanced esophageal cancer.

**Methods:**

Clinical information of patients with recurrence/metastasis and death after radical resection of esophageal cancer at our hospital between January 1, 2005, and December 31, 2015, were retrospectively collected and followed up. Postoperative recurrence-free survival time, postrelapse survival time, and overall survival time were compared among the metabolic-associated, organ failure-associated, and anastomotic recurrence-associated mortality groups.

**Results:**

Five hundred and ninety-five qualified patients were retrieved, including 456 males and 139 females, with an average age of 58 ± 7.56 years. There were 57 cases of TNM-1 stage, 131 cases of TNM-2 stage, 365 cases of TNM-3 stage, and 42 cases of TNM-4 stage. There were 547 cases of squamous cell cancer and 48 cases of nonsquamous cell cancer. There were significant differences in age (*p* < 0.01), tumor location (*p* < 0.01), and lymph node metastasis (*p* = 0.04), recurrence type (*p* < 0.01) by one-way ANOVA, and recurrence-free survival (*p* = 0.02) and postrecurrence survival (*p* < 0.01) by Kaplan-Meier survival curve analysis among the three main death causes.

**Conclusions:**

Age, tumor location, and lymph node metastasis were significantly different among metabolic-associated, organ failure-associated, and anastomotic recurrence-associated mortality of recurrent EC patients.

## 1. Introduction

Esophageal cancer (EC) is one of the most common malignant upper gastrointestinal tumors and ranks the fourth cause of cancer-related mortality in China [1]. In 2017, there were 234,624 new cases of EC and 212,586 new deaths due to EC in China [2]. Risk factors of EC include smoking, heavy drinking, nitrosamine and certain mold/fungi, gastroesophageal reflux disease (GERD), and Barrett's esophagus. In EC cases at early-mid clinical stages or above, surgery with postoperative adjuvant chemotherapy or radiotherapy is the most accepted treatment. However, after surgery and adjuvant therapy, 30%-40% of cases will still develop lymph node metastasis within 2 years, with poor treatment response and a median survival of 7 only months [1]. Previous studies have shown that postoperative lymph node metastasis and other related factors affect the postoperative recurrence and metastasis rates, but the characteristic patterns of recurrence, metastasis, and cancer-related death in patients with EC after radical resection and postoperative adjuvant chemotherapy or radiotherapy remain unclear. Therefore, we retrospectively collected patients with recurrence/metastasis after radical resection of esophageal cancer at our hospital and analyzed the relationship between patients' clinical characteristics and their recurrence/metastasis patterns and death patterns, in order to provide evidence to clarify the disease process of advanced EC.

The article "Posttreatment Recurrence and Death Patterns in Patients with Advanced Esophageal Cancer" was published in 2022. Journal: Dis Markers.

## 2. Materials and Methods

### 2.1. Population

The present study was approved by the ethics committee of our hospital. Patients' information with posttreatment recurrence of EC [3] who were treated at our hospital from January 1, 2005, to December 31, 2015, was retrospectively collected. The following are the inclusion criteria: thoracic EC cases [4] and received esophagectomy, upper and lower stumps negative for cancer lesions, number of lymph nodes collected ≥16; and having complete postoperative adjuvant therapy information. The following are the exclusion criteria: those who suffered from other malignant tumors at the same time or after EC or those who were lost to follow-up for more than 6 months.

### 2.2. Follow-up Items

The requirement for follow-up within 2 years after operation included reexamination of chest and upper abdominal CT and esophagography every 3 (±1) months to determine the status of regional lymph nodes and anastomotic stoma, then every 6 months between 2-5 years after operation for similar items. According to the 8th edition of NCCN TNM staging standard for esophageal cancer [4], postoperative recurrence-free survival was defined as the time after surgery to the time of tumor recurrence or disease progression based on the pathology report during follow-up. Postrelapse survival time was defined as the time from the diagnosis of relapse to death. The definition of recurrence pattern is as follows: recurrence of anastomotic stoma refers to reexamination of new organisms and biopsy confirmed by biopsy; lymph node recurrence referred to reexamination of CT scan showing new enlarged lymph nodes with a short diameter greater than 1 cm. The definition of main death modes is as follows: metabolic disorder-related death was defined as death caused by chronic low serum protein, electrolyte imbalance, and other symptoms of cachexia; organ failure-related death was defined as death caused by clear diagnosis of heart, lung, liver, or multiple organ failure; anastomotic-related death was defined as death due to anastomotic-site fistula-induced infection or major bleeding. Adjuvant chemotherapy was defined as receiving at least once of platinum-containing combination chemotherapy after surgery.

The article "Posttreatment Recurrence and Death Patterns in Patients with Advanced Esophageal Cancer" was published in 2022. Journal: Dis Markers.

### 2.3. Statistics

SPSS 24.0 software (SPSS Inc., Chicago, USA) was used to analyze the differences in survival time and survival rate of patients. The difference in median recurrence-free survival time between the two groups was analyzed by a *t* test, while the difference in median recurrence-free survival time between multiple groups was analyzed by one-way ANOVA, and the difference in survival rate was analyzed by a chi-square test. Correlation analysis was performed using Pearson's correlation coefficient analysis. Differences in survival curves were analyzed using Log-Rank analysis within Kaplan-Meier survival curve. A two-tailed *p* value less than 0.05 was considered to be statistically significant.

## 3. Results

### 3.1. General Conditions of Enrolled Patients

There were 5613 EC cases who received esophagectomy at our center from January 1, 2005, to December 31, 2015. Seven hundred and six patients had recurrence, and 595 cases were included for analysis, including 25 cases of rare causes of death and 570 cases of main causes of death (320 cases for metabolic-associated deaths, 135 cases for organs failure-associated deaths, and 115 cases of anastomotic recurrence-associated deaths, Figure 1). There were 456 males and 139 females, with an average age of 58 ± 7.56 years. There were 57 cases of TNM-1 stage, 131 cases of TNM-2 stage, 365 cases of TNM-3 stage, and 42 cases of TNM-4 stage. There were 547 cases of squamous cell cancer and 48 cases of nonsquamous cell cancer (Table 1).

### 3.2. Metastasis Characteristics of Died Patients due to Recurrence

In a detailed analysis of the cause of mortality in the metabolic-associated category, there were 190 cases of extensive lymph node metastasis, 45 cases of cachexia, 40 cases of bone metastasis, 29 cases of liver metastasis, and 16 cases of rare metastasis. In the organ failure-associated category, there were 106 cases due to respiratory failure, 21 cases due to multiple organ failure, 6 cases due to circulatory failure, and 2 cases of hepatic failure. In the anastomotic recurrence-associated category, there were 95 cases of hematemesis and 20 cases of fistula. There were also 5 cases of brain/meningeal metastasis, 4 cases of serious infections, and 16 cases of noncancer mortality (Table 2). Among the three main death causes, there were significant differences in recurrence type, recurrence-free survival, and postrecurrence survival among the three main death causes (*p* < 0.05 for all comparisons, Table 3).

The article "Posttreatment Recurrence and Death Patterns in Patients with Advanced Esophageal Cancer" was published in 2022. Journal: Dis Markers.

### 3.3. Clinical Characteristics of Patients due to Different Death Causes

There were no significant differences in gender (*p* = 0.53), tumor size (*p* = 0.75), tumor stage (*p* = 0.86), pathological types (*p* = 0.83), differentiation grade (*p* = 0.18), location of anastomoses (*p* = 0.07), R0 resection (*p* = 0.92), or adjuvant therapy (*p* = 0.93), but there are significant differences in age (*p* < 0.01), tumor location (*p* < 0.01), and lymph node metastasis (*p* = 0.04) among the three main death cause groups, e.g., metabolic-associated, organ failure-associated, and anastomotic recurrence-associated (Table 4). According to the Kaplan-Meier survival curve, there were significant differences in recurrence-free survival (*p* = 0.02) and postrecurrence survival (*p* < 0.01), but not in overall survival (*p* = 0.10) among the three main death cause groups (Figures 2–4).

## 4. Discussion

Many biomarkers for EC have been reported [5–7]. However, some studies reported lymph node metastases patterns at the time of surgery [8, 9], and to attribute the recurrence/metastasis patterns and death patterns of advanced EC to patients' clinical characteristics is still a big challenge. In this study, we retrospectively collected 595 cases who died due to recurrence of EC and analyzed the recurrence and death patterns. We found that metabolic-associated causes (53.8%) accounted for the majority of death, followed by organ failure-associated (22.7%) and anastomotic recurrence-associated (19.3%) causes.

Compared with a recent study by Sohda et al. [10], which contained 307 EC cases (197 nonrecurrence cases and 110 recurrence cases) from Japan, more EC-recurrent patients (*n* = 595) were enrolled in our study. Their findings that 92% recurrent were observed in less than 2 years after radical esophagectomy have a similar trend as our findings, which was much higher than the 30-40% by Chinese surveillance [1]. The difference between their and our findings might be due to the difference in the composition of pathological types (squamous cell: 83.4% in their study vs. 91.9% in our study), age (mean: 65.2 years old in their study vs. 58 years old in our study) [11, 12] and living environment and habits [13–15]. They also found that patients with lymph node metastasis survived significantly longer than those metastasized to other organs and patients after surgical or additional postoperative chemotherapy lived longer than those who received other treatments. Due to the difference in study design, we could not validate the above two findings in our cohort of EC patients.

The article "Posttreatment Recurrence and Death Patterns in Patients with Advanced Esophageal Cancer" was published in 2022. Journal: Dis Markers.

In another study by Yang et al. [16], 95 recurrent EC patients was analyzed. Among them, 4 (4.2%) were local-only, 40 (42.1%) were regional-only, 44 (46.3%) were hematogenous-only, and 7 (7.4%) were combined recurrences, while in our study, we included all dead patients and divided the recurrence pattern into metabolic-associated, organ failure-associated, and anastomotic recurrence-associated groups, which was more detailed and cause-attributable. They also found that cervical lymph nodes were the most frequent sites of regional recurrence, whereas the lung was the most hematogenous recurrence site. Their median recurrence-free interval was 12.1 months (versus 12 months in the metabolic-associated group, 14.5 months in the organ failure-associated group, and 16 months in the anastomotic recurrence-associated group in our study). In their study, tumor in the upper esophagus, larger tumor length, and positive lymph nodes were independent risk factors for recurrence. In contrast, we found that age, tumor location, and positive lymph nodes were significantly different among the three main death cause groups. Again, our findings among the dead patients drew a much closer picture of the death pattern based on more enrolled dead cases. It is also interesting to note that some clinical conditions, such as hepatitis, HPV, inflammation, or hypoxia, might affect the development or recurrence of EC [17–20].

In conclusion, based on our relative large enrolled number of patients, age, tumor location, and lymph node metastasis were significantly different among metabolic-associated, organ failure-associated, and anastomotic recurrence-associated mortality of recurrent EC patients.

## Figures and Tables

**Figure 1:** Flow chart of patient screening.

**Figure 2:** Kaplan-Meier survival curve of recurrence-free survival among the metabolic-associated, organ failure-associated, and anastomotic recurrence-associated mortality groups.

**Figure 3:** Kaplan-Meier survival curve of post-recurrence survival among the metabolic-associated, organ failure-associated, and anastomotic recurrence-associated mortality groups.

**Figure 4:** Kaplan-Meier survival curve of overall survival among the metabolic-associated, organ failure-associated, and anastomotic recurrence-associated mortality groups.

**Table 1:** Basic characteristics of enrolled patients (*n* = 595).

	Number	Rate%
Gender		
Male	456	76.6
Female	139	23.4
Age	58 ± 7.56	
Tumor location		
Upper	66	11.1
Middle	409	68.7
Lower	120	20.2
Tumor size	5 ± 2.05	
TNM stage		
1	57	9.6
2	131	22
3	365	61.3
4	42	7.1
Lymph node metastasis		
Negative	272	45.7
Positive	323	54.3
Pathological types		
Squamous cell cancer	547	91.9
Nonsquamous cell cancer	48	8.1
Differentiation grade		
Well	324	54.4
Poor	264	44.4
Undifferentiated	7	1.2
Location of anastomoses		
Neck	90	15.1
On the arch aor	460	77.3
Under the arch aor	45	7.6
R0 resection		
Yes	540	90.7
No	55	9.3
Stump pathological grade		
Normal	540	90.7
Atypical hyperplasia	22	3.7
Carcinoma	33	5.6

The article "Posttreatment Recurrence and Death Patterns in Patients with Advanced Esophageal Cancer" was published in 2022. Journal: Dis Markers.

**Table 2:** Metastasis characteristics of died patients due to recurrence.

Cause of mortality	Number	Rate (%)
Metabolic-associated	320	53.8
Extensive lymph node metastasis	190	31.9
Cachexia	45	7.6
Bone metastasis	40	6.7
Liver metastasis	29	4.9
Rare metastasis	16	2.7
Organ failure-associated	135	22.7
Respiratory failure	106	17.8
Multiple organ failure	21	3.5
Circulatory failure	6	1
Hepatic failure	2	0.3
Anastomotic recurrence-associated	115	19.3
Hematemesis	95	15.9
Fistula	20	3.4
Brain/meningeal metastases	5	0.8
Serious infections	4	0.7
Non-cancer mortality	16	2.7

**Table 3:** Recurrence type and survival of 3 main death causes.

	Cause of mortality (*n*)			*p* value
	Metabolic-associated	Organ failure-associated	Anastomotic recurrence-associated	
Recurrence type (*n*)				<0.01
Anastomosis associated	11	8	58	
Local lymph node metastasis	243	109	53	
Distant lymph node metastasis	66	18	4	
Recurrence-free survival (months, mean ± SD)	12 ± 17.28	14.5 ± 23.11	16 ± 32.34	0.02
Post-recurrence survival (months, mean ± SD)	10 ± 11.02	16 ± 13.31	11 ± 12.7	<0.01
Overall survival (months, mean ± SD)	24 ± 21.27	32 ± 26.48	26 ± 36.36	0.10

**Table 4:** Clinical characteristics of patients due to different death causes.

	Cause of mortality			*p* value
	Metabolic-associated	Organ failure-associated	Anastomotic recurrence-associated	
Gender (*n*)				0.53
Male	245	100	92	
Female	75	35	23	
Age (year, mean ± SD)	57 ± 7.01	59 ± 7.9	58 ± 7.94	<0.01
Tumor location (*n*)				<0.01
Upper	27	14	20	
Middle	221	103	67	
Lower	72	17	28	
Tumor size (cm, mean ± SD)	5 ± 1.89	5 ± 2.2	5 ± 2.32	0.75
Tumor stage (*n*)				0.86
1	34	13	8	
2	71	32	25	
3	199	79	69	
4	16	11	13	
Lymph node metastasis (*n*)				0.04
Negative	137	62	64	
Positive	183	73	51	
Pathological types (*n*)				0.83
Squamous cell cancer	295	125	108	
Nonsquamous cell cancer	25	10	7	
Differentiation grade (*n*)				0.18
Well	162	81	66	
Poor	157	51	47	
Undifferentiated	1	3	2	
Location of anastomoses (*n*)				0.07
Neck	42	17	26	
On the arch	249	115	79	
Under the arch	29	3	10	
R0 resection (*n*)				0.92
Yes	292	120	105	
No	28	15	10	
Adjuvant therapy (*n*)				0.93
No	134	55	46	
Chemotherapy	149	63	52	
Radio/chemo	37	17	17	

The article "Posttreatment Recurrence and Death Patterns in Patients with Advanced Esophageal Cancer" was published in 2022. Journal: Dis Markers.

## Data Availability

The data used to support the findings of this study were supplied by the Institutional Ethnics Committee of the Fourth Hospital of Hebei Medical University under license and so cannot be made freely available. Requests for access to these data should be made to Dr. Jidong Zhao (e-mail: zjd2016@hebmu.edu.cn).

## References

[1] NHC of the People (2019). Chinese guidelines for diagnosis and treatment of esophageal carcinoma 2018 (English version). *Chinese Journal of Cancer Research*.

[2] Yang S., Lin S., Li N. (2020). Burden, trends, and risk factors of esophageal cancer in China from 1990 to 2017: an up-to-date overview and comparison with those in Japan and South Korea. *Journal of Hematology & Oncology*.

[3] Ekeke C. N., Chan E. G., Fabian T., Villa-Sanchez M., Luketich J. D. (2021). Recommendations for surveillance and management of recurrent esophageal cancer following endoscopic therapies. *The Surgical Clinics of North America*.

[4] Rice T. W., Patil D. T., Blackstone E. H. (2017). 8th edition AJCC/UICC staging of cancers of the esophagus and esophagogastric junction: application to clinical practice. *Annals of cardiothoracic surgery*.

[5] Chen C., Zhao J., Liu J. N., Sun C. (2021). Mechanism and role of the neuropeptide LGI1 receptor ADAM23 in regulating biomarkers of ferroptosis and progression of esophageal cancer. *Disease Markers*.

[6] Dai X., Sun X., Wu Y. (2022). Site-specifichypermethylation of SST 1stExon as a biomarker for predicting the risk of gastrointestinal tract cancers. *Disease Markers*.

[7] Wang P., Chen Y., Zheng Y., Fu Y., Ding Z. (2021). Identification of epithelial-mesenchymal transition- (EMT-) related LncRNA for prognostic prediction and risk stratification in esophageal squamous cell carcinoma. *Disease Markers*.

[8] Harrington C. A., Carr R. A., Hsu M. (2022). Patterns and influence of nodal metastases after neoadjuvant chemoradiation and R0 resection in esophageal adenocarcinoma. *The Journal of Thoracic and Cardiovascular Surgery*.

[9] Wen J., Chen J., Chen D. (2021). Comprehensive analysis of prognostic value of lymph node classifications in esophageal squamous cell carcinoma: a large real-world multicenter study. *Therapeutic Advances in Medical Oncology*.

[10] Sohda M., Yoshida T., Nakazawa N. (2021). Comparative study on recurrence pattern and treatment method after radical esophagectomy for esophageal cancer. *The Journal of Medical Investigation*.

[11] Dezube A. R., Cooper L., Mazzola E. (2022). Long-term outcomes following esophagectomy in older and younger adults with esophageal cancer. *Journal of Gastrointestinal Surgery*.

The article "Posttreatment Recurrence and Death Patterns in Patients with Advanced Esophageal Cancer" was published in 2022. Journal: Dis Markers.

[12] Chen Y., Yang C., Li N. (2022). Effects of population aging on the mortality burden of related cancers in urban and rural areas of China, 2004-2017: a population-based study. *Cancer biology & medicine*.

[13] Li Y., Xu J., Gu Y., Sun X., Dong H., Chen C. (2022). The disease and economic burdens of esophageal cancer in China from 2013 to 2030: dynamic cohort modeling study. *JMIR Public Health and Surveillance*.

[14] Fahey P. P., Page A., Astell-Burt T., Stone G. (2021). Imputing pre-diagnosis health behaviour in cancer registry data and investigating its relationship with oesophageal cancer survival time. *PLoS One*.

[15] Park S. Y., Kim D. J. (2021). Esophageal cancer in Korea: epidemiology and treatment patterns. *Journal of Chest Surgery*.

[16] Yang Y., Zhang H., Li B. (2022). Patterns of recurrence after robot-assisted minimally invasive esophagectomy in esophageal squamous cell carcinoma. *Seminars in Thoracic and Cardiovascular Surgery*.

[17] Bekmukhambetov Y. Z., Mynbaev O. A., Tinelli A. (2018). Human papillomavirus related issues in western Kazakhstan: protocol for a comprehensive study. *Russian Open Medical Journal*.

[18] Vásquez-Vivar J., Shi Z., Tan S. (2022). Tetrahydrobiopterin in cell function and death mechanisms. *Antioxidants & Redox Signaling*.

[19] Shi Z., Vasquez-Vivar J., Luo K. (2019). Ascending lipopolysaccharide-induced intrauterine inflammation in near-term rabbits leading to newborn neurobehavioral deficits. *Developmental Neuroscience*.

[20] Li X. M., Ma L., Yang Y. B., Shi Z. J., Zhou S. S. (2005). Prognostic factors of fulminant hepatitis in pregnancy. *Chinese Medical Journal*.

